The article "LINC00265 targets miR-382-5p to regulate SAT1, VAV3 and angiogenesis in osteosarcoma" was retracted in 2025. Reasons: duplicated images; signs of a paper mill; concerns about the images.

# LINC00265 targets miR-382-5p to regulate SAT1, VAV3 and angiogenesis in osteosarcoma

**DOI:** 10.18632/aging.103762

**Published:** 2020-08-14

**Authors:** Ying Xiao, Chunling Li, Hongyue Wang, Yijun Liu

**Affiliations:** 1 Department of Operating Center, The First Hospital of Jilin University, Changchun 130000, Jilin, China; 2 Department of Nephrology, The First Hospital of Jilin University, Changchun 130000, Jilin, China; 3 Department of Orthopaedics, The First Hospital of Jilin University, Changchun 130000, Jilin, China

**Keywords:** angiogenesis, vasculogenic mimicry, LINC00265, miR-382-5p, spermidine/spermine N1-acetyltransferase-1

## Abstract

We explored the mechanism by which LINC00265 regulates angiogenesis of osteosarcoma cells via the miR-382-5p/spermidine/spermine *N1*-acetyltransferase-1 (SAT1) and miR-382-5p/vav guanine nucleotide exchange factor 3 (VAV3) axis. Cell scratch assay, Transwell assay and tube formation assay were applied to detect cell migration, invasion and tube formation abilities. The effects of LINC00265 targeting miR-382-5p in osteosarcoma in vivo were studied using a tumour-burden assay. A total of 70 genes potentially involved in osteosarcoma angiogenesis were identified, and a Gene Ontology (GO) analysis found that SAT1 and VAV3 were closely related to angiogenesis. Bioinformatics analysis and clinical experiments confirmed that LINC00265, SAT1 and VAV3 were overexpressed in osteosarcoma and related to a poor prognosis, whereas miR-382-5p was downregulated and associated with a poor prognosis. It was confirmed that LINC00265 promoted the proliferation, migration, invasion and angiogenesis of osteosarcoma cells by targeting miR-382-5p to mediate SAT1 and VAV3. Collectively, LINC00265 might promote proliferation, migration, invasion and angiogenesis by targeting miR-382-5p/SAT1 and miR-382-5p/VAV3 in osteosarcoma.

## INTRODUCTION

Osteosarcoma is a malignant tumour originating from mesenchymal cells and has an incidence of approximately 3 % [1]. Osteosarcoma is more likely to occur at the ends of long bones, and the incidence of osteosarcoma in males is higher than that in females [2, 3]. Osteosarcoma progresses rapidly and has high morbidity and mortality [4, 5]. To date, the main treatments for osteosarcoma include surgery, chemotherapy, immunotherapy and gene therapy [6–8]. However, the high metastatic ability and drug resistance of osteosarcoma are the main causes of poor prognosis [9, 10].

MicroRNA (miRNA) can cause message RNA (mRNA) degradation or translational inhibition by targeting the 3' untranslated region (UTR) of mRNA, [11, 12]. Long noncoding RNA (lncRNA) is a type of RNA that is more than 200 nucleotides in length but does not have protein translation capabilities [13–15]. LncRNA has the role of regulating epigenetics by activating or interfering with transcription [16, 17]. LncRNA forms complementary double-strands with the transcripts of exon genes, interfering with mRNA splicing, and then produces different forms of splicing to affect gene expression [18]. LncRNA can also target microRNA (miRNA) and act as a sponge, thereby regulating the process of miRNA targeting mRNA [19–21]. LncRNA can target miRNA by competing endogenous RNA (ceRNA) [22]. MiRNA can cause messenger RNA (mRNA) degradation or translational inhibition by targeting the 3' untranslated region (UTR) of mRNA [11, 12]. The role of lncRNA-miRNA-mRNA in the regulation of cancers is gradually being discovered [23–25]. However, the number of RNAs is large, and bioinformatics analysis helps to screen for meaningful genes [26, 27]. LINC00265 is a newly discovered tumour-associated lncRNA that has a significant promoting effect on colorectal cancer [28], acute myeloid leukaemia [29] and lung adenocarcinoma [30]. However, the role and mechanism of LINC00265 in osteosarcoma is still unclear. The lncRNA-miRNA-mRNA network is relatively complex, and the use of bioinformatics can help identify key lncRNA, miRNA, and target genes. The genomic spatial event (GSE) database contains high-throughput gene expression data submitted by research institutions from various countries to the National Center for Biotechnology Information (NCBI), and this database can help to identify key lncRNAs.

In this paper, using a bioinformatics analysis, we found that LINC00265, spermidine/spermine *N1*-acetyltransferase-1 (SAT1) and vav guanine nucleotide exchange factor 3 (VAV3) were overexpressed in osteosarcoma, showed a positive correlation with osteosarcoma, and were associated with a poor prognosis in osteosarcoma patients. Based on this, we revealed a mechanism by which LINC00265 promoted migration, invasion and angiogenesis of osteosarcoma cells via miR-382-5p/SAT1 or/VAV3. These findings may provide new avenues for the discovery of strategies for osteosarcoma treatment.

## RESULTS

### Analysis of GEO data

GSE119975 contained 3 osteosarcoma samples with vasculogenic mimicry and 3 osteosarcoma samples without vasculogenic mimicry. The samples passed the correction (Figure 1A). There were 529 differentially expressed lncRNAs, of which 274 lncRNAs were downregulated and 255 were upregulated (Figure 1B). There were 91 differentially expressed miRNAs, of which 4 miRNAs were downregulated and 87 were upregulated (Figure 1C). There were 2,214 differentially expressed genes, of which 1378 were downregulated and 836 were upregulated (Figure 1D). Among them, LINC00265 and LINC00342 were significantly overexpressed in the vasculogenic mimicry osteosarcoma cell line. To date, there is little data on LINC00265 and LINC00342, which aroused our interest.

**Figure 1:** **Bioinformatics analysis.** (**A**) Correction of the GSE119975 gene chip. (**B–D**) Differential expression analysis of the lncRNA, miRNA and mRNA of GSE119975. (**E**) Correction of the GSE12865 gene chip. (**F, G**) Differential expression analysis of the miRNA and gene of GSE12865. (**H, I**) Gene Ontology (GO) analysis of 70 genes overexpressed by GSE119975 and GSE12865.

GSE12865 contained 2 normal tissue samples and 12 osteosarcoma tissue samples and the samples were corrected (Figure 1E). There were 27 differentially expressed miRNAs, of which 17 were downregulated and 10 were upregulated (Figure 1F). There were 4410 differentially expressed genes, of which 3,088 were downregulated and 1,322 were upregulated (Figure 1G).

The upregulated genes in GSE119975 and GSE12865 were analysed to obtain the intersection of 70 genes (Figure 3A). These 70 genes were analysed using Gene Ontology (GO), which showed that they were enriched in 16 pathways. The 70 genes were primarily enriched in the angiogenesis pathway and G-protein coupled receptor signalling pathway, both of which belong to the category of biological processes (Figure 1H, 1I). Five genes were included in the angiogenesis pathway: NRP2, PIK3CG, SAT1, VAV3 and ANGPT2. PIK3CG was also in the G-protein coupled receptor signalling pathway. SAT1 and VAV3 were primarily involved in angiogenesis, so we chose PIK3CG, SAT1 and VAV3 as research targets.

### Expression characteristics of LINC00265, LINC00342, PIK3CG, SAT1, and VAV3 in osteosarcoma patients and their relationship with prognosis

The results of the qPCR showed that LINC00265, LINC00342, PIK3CG, SAT1, and VAV3 were overexpressed in osteosarcoma patients (Figure 2A–2E). In osteosarcoma tissues, the expression level of LINC00265 showed a significant positive correlation with SAT1 and VAV3; LINC00342 was not significantly correlated with the genes (Figure 2F–2H). A survival analysis showed that high levels of LINC00265, PIK3CG, SAT1 and VAV3 were associated with a poor prognosis in patients with osteosarcoma (Figure 2I–2M). Immunohistochemical staining and Western blot results also showed that SAT1 and VAV3 were overexpressed in osteosarcoma tissues.

**Figure 2:** **Expression characteristics of LINC00265, LINC00342, PIK3CG, SAT1 and VAV3 in osteosarcoma patients and the relationship with prognosis.** (**A–E**) Expression levels of LINC00265, LINC00342, PIK3CG, SAT1 and VAV3 in osteosarcoma and adjacent tissues. (**F–H**) Correlation between lncRNA and mRNA expression levels. **(I–M**) The relationship between LINC00265, LINC00342, PIK3CG, SAT1 and VAV3 levels and prognosis. (**N**, **O**) Expression characteristics of SAT1 and VAV3 proteins in osteosarcoma tissues.

### LINC00265 regulates SAT1 and VAV3 by targeting miR-382-5p

We predicted the downstream miRNA targets of LINC00265 through the website and predicted upstream miRNAs that might induce SAT1 and VAV3. The predicted results of LINC00265, SAT1 or VAV3 were combined with the downregulated miRNAs in GSE12865 to obtain miRNAs held in common. The results showed that LINC00265 and SAT1 or VAV3 each had one miRNA, which was miR-382-5p (Figure 3B, 3C). LINC00265 targeted miRNA, PIK3CG targeted miRNA, and for miRNAs that were downregulated, there was no intersecting miRNA. The results of clinical studies showed that miR-382-5p was underexpressed in osteosarcoma and negatively correlated with LINC00265, SAT1 and VAV3 (Figure 3D–3G). A survival analysis also showed that low expression of miR-382-5p was associated with poor pre-exposure (Figure 3H). This suggested that in osteosarcoma, LINC00265 might promote SAT1 and VAV3 by targeting miR-382-5p and thus participate in the development and progression of osteosarcoma.

**Figure 3:** **LINC00265 regulated SAT1 and VAV3 by targeting miR-382-5p.** (**A**) The Venn diagram of genes upregulated in GSE119975 and GSE12865. (**B**, **C**) The Venn diagram of upstream miRNAs for SAT1 and VAV3, downstream target miRNAs of LINC00265, and downregulated miRNAs in GSE119975 and GSE12865. (**D**) Expression characteristics of miR-382-5p in osteosarcoma tissues. (**E–G**) Correlation analysis of miR-382-5p and LINC00265, SAT1 or VAV3. (**H**) The relationship between miR-382-5p and prognosis.

We next examined the expression levels of LINC00265, miR-382-5p, SAT1, and VAV3 in human osteoblasts and osteosarcoma cell lines. The results showed that in the osteosarcoma cell line, LINC00265, SAT1, and VAV3 were overexpressed, and miR-382-5p was downregulated. These trends were most prominent in the 143B and U2OS cell lines (Figure 4A–4C). A luciferase assay and cell experiments showed that LINC00265 targeted miR-382-5p and miR-382-5p targeted SAT1 and VAV3 (Figure 4D–4J). This indicated that miR-382-5p could target SAT1 and VAV3, whereas miR-382-5p was sponged by LINC00265.

**Figure 4:** **Luciferase assay was used to validate targeting relationships**. (**A-C**) Expression levels of LINC00265, miR-382-5p, SAT1 and VAV3 in osteosarcoma cells and osteoblasts. (**D**) Transfection efficiency of OE-LINC00265 and sh-LINC00265. (**E, F**) Luciferase assay confirmed that LINC00265 targeted miR-382-5p. (**G**) Transfection efficiency of miR-382-5p inhibitor and miR-382-5p mimic. (**H-J**) Luciferase assay confirmed that miR-382-5p targeted SAT1 and VAV3. ^*^P < 0.05 vs. sh-NC or inhibitor-NC group; ^#^P < 0.05 vs. OE-NC or mimic-NC group.

### MiR-382-5p targets SAT1 and VAV3 to inhibit osteosarcoma cell proliferation, migration, invasion and tube formation

To analyse the effects of miR-382-5p targeting SAT1 on osteosarcoma cells, the 143B and U2OS cell lines were divided into four groups: sh-NC+inhibitor-NC, sh-NC+inhibitor, sh-SAT1+inhibitor and sh-SAT1+inhibitor-NC. The transfection efficiency was determined by qPCR experiments, and it was verified that in osteosarcoma cell lines, the inhibitor could promote the expression of SAT1 mRNA and protein (Figure 5A–5C). Downregulation of miR-382-5p promoted cell proliferation, migration, invasion, and tube formation. Knockdown SAT1 inhibited cell proliferation, migration, invasion, and tube formation and reversed the proliferative effects of the miR-382-5p inhibitor (Figure 5D, 5E).

**Figure 5:** **MiR-382-5p targets SAT1 to regulate osteosarcoma cell proliferation, migration, invasion and tube formation**. (**A**) The expression level of miR-382-5p in each group. (**B**, **C**) The expression level of SAT1 mRNA and protein in each group. (**D**, **E**) CCK-8 and colony formation assays were used to detect cell viability and proliferation. (**F**, **G**) Wound healing and Transwell assays were applied to detect cell migration and invasive ability. (**H**) The tube production capacity of the cells was detected using tube formation assay. ^*^P < 0.05 vs. sh-NC+inhibitor-NC group; ^#^P < 0.05 vs. sh-NC+inhibitor group.

To analyse the effects of miR-382-5p targeting VAV3 on osteosarcoma cells, the 143B and U2OS cell lines were divided into four groups: sh-NC+inhibitor-NC, sh-NC+inhibitor, sh-VAV3+inhibitor and sh-VAV3+inhibitor-NC. The results also showed that downregulation of VAV3 inhibited the proliferation, migration, invasion, and tube formation of osteosarcoma cells, and partially reversed the effects of the miR-382-5p inhibitor (Figure 6A–6H).

**Figure 6:** **MiR-382-5p targets VAV3 to regulate osteosarcoma cell proliferation, migration, invasion and tube formation.** (**A**) The expression level of miR-382-5p in each group. (**B**, **C**) The expression level of VAV3 mRNA and protein in each group. (**D**, **E**) CCK-8 and colony formation assays were used to detect cell viability and proliferation. (**F**, **G**) Wound healing and Transwell assays were applied to detect cell migration and invasive ability. (**H**) The tube production capacity of the cells was detected using the tube formation assay. ^*^P < 0.05 vs. sh-NC+inhibitor-NC group; ^#^P < 0.05 vs. sh-NC+inhibitor group.

These results demonstrated that SAT1 and VAV3 promoted metastasis and tube formation in osteosarcoma and that they were targeted by miR-382-5p.

### LINC00265 promotes osteosarcoma cell metastasis and tube formation by targeted regulation of miR-382-5p/SAT1 and miR-382-5p/VAV3

To further study the regulatory mechanism of LINC00265, we divided the 143B and U2OS cell lines into four groups: sh-NC+inhibitor-NC, sh-LINC00265+inhibitor-NC, sh-LINC00265+inhibitor and sh-NC+inhibitor-NC. The results showed that the miR-382-5p inhibitor had no significant effect on the level of LINC00265 (Figure 7A). Downregulation of LINC00265 significantly promoted miR-382-5p levels and inhibited the mRNA and protein levels of SAT1 and VAV3, and the miR-382-5p inhibitor partially reversed the inhibitory effects of sh-LINC00265 on SAT1 and VAV3 (Figure 7B–7F). Further experimentation also confirmed that downregulation of LINC00265 could inhibit cell viability, migration, invasion, and tube formation of osteosarcoma cells, and the miR-382-5p inhibitor could partially reverse the effects of LINC00265 on cells. These results showed that LINC00265 could promote osteosarcoma cell metastasis and tube formation through targeted regulation of miR-382-5p/SAT1 and miR-382-5p/VAV3.

**Figure 7:** **LINC00265 regulated osteosarcoma cell metastasis and tube formation by targeted regulation of miR-382-5p/SAT1 and miR-382-5p/VAV3**. (**A**, **B**) The expression level of LINC00265 and miR-382-5p in each group. (**C–F**) The expression level of SAT1 and VAV3 mRNA and protein in each group. (**G**, **H**) CCK-8 and colony formation assays were used to detect cell viability and proliferation. (**I**, **J**) Wound healing and Transwell assays were applied to detect cell migration and invasive ability. (**K**) The tube production capacity of the cells was detected using the tube formation assay. ^*^P < 0.05 vs. sh-NC+inhibitor-NC group; ^#^P < 0.05 vs. sh-LINC00265+inhibitor-NC group.

### LINC00265 promotes osteosarcoma growth by regulating miR-382-5p/SAT1 and miR-382-5p/VAV3

To further analyse the effects and mechanism of LINC00265 on osteosarcoma, we performed a subcutaneous tumour formation experiment in nude mice. The results showed that the tumour weight and volume of the sh-LINC00265+inhibitor-NC group were significantly lower than those of the sh-NC+inhibitor-NC group, the tumour weight and volume of the sh-NC+inhibitor group were significantly increased, and the tumour weight and volume of the sh-LINC00265+inhibitor group was significantly higher than those of the sh-LINC00265+inhibitor-NC group (Figure 8A, 8B). Further studies showed that downregulation of LINC00265 inhibited SAT1 and VAV3 mRNA and protein levels in tumour tissues, whereas downregulation of miR-382-5p partially reversed the effects of downregulation of LINC00265 on SAT1 and VAV3 expression (Figure 8C–8F). Similar results were obtained in the immunohistochemistry experiments, and it was found that SAT1 and VAV3 were primarily expressed in the nucleus and cytoplasm (Figure 8G, 8H). This suggested that LINC00265 could promote osteosarcoma growth by regulating miR-382-5p/SAT1 and miR-382-5p/VAV3.

**Figure 8:** **LINC00265 regulated osteosarcoma growth by regulating miR-382-5p/SAT1 and miR-382-5p/VAV3**. (**A**, **B**) Effects of LINC00265 and miR-382-5p on tumour mass and volume. (**C**, **D**) Effects of LINC00265 on the expression levels of SAT1 and VAV3 mRNAs by targeting miR-382-5p. (**E**, **F**) Effects of LINC00265 on the expression levels of SAT1 and VAV3 by targeting miR-382-5p. (**G**, **H**) Immunohistochemistry staining was used to detect the expression of SAT1 and VAV3 proteins in tumour tissues. ^*^P < 0.05 vs. sh-NC+inhibitor-NC group; ^#^P < 0.05 vs. sh-LINC00265+inhibitor-NC group.

## DISCUSSION

In this study, we discovered the role of LINC00265, SAT1 and VAV3 in osteosarcoma through bioinformatics and analysed the mechanism by which LINC00265 promotes the migration, invasion and tube formation of osteosarcoma cells via miR-382-5p targeting of SAT1 and VAV3. The high metastasis and recurrence rate of osteosarcoma is one of the primary factors affecting the prognosis of patients [31]. Tumour cells acquire migration capacity and are transferred to various parts of the body through blood vessels and lymphatic vessels [32, 33]. Vasculogenic mimicry is a new form of tumour tissue angiogenesis that promotes angiogenesis in tumour tissues, increases the supply of oxygen and nutrients to tumour tissues, and provides a basis for tumour cell metastasis [34–36]. Studies have shown that vasculogenic mimicry is a contributing factor to the poor prognosis of malignant invasive tumours [37, 38]. Therefore, we analysed the GSE119975 data using a differential analysis. The GSE119975 data contained two groups—non-vasculogenic mimicry cells and vasculogenic mimicry cells—and the difference in gene expression between the two groups was compared in a microarray. It was found that LINC00265 and LINC00342 were significantly overexpressed in the vasculogenic mimicry osteosarcoma cell line. Bioinformatics analyses show that LINC00265 is overexpressed in colorectal cancer and positively correlated with the level of the oncogene [39]. LINC00265 may participate in the occurrence and development of lung adenocarcinoma through the mechanism of ceRNA [30]. One study found that LINC00342 is upregulated in patients with non-small cell lung cancer, and its level is positively correlated with lymph node metastasis, tumour metastasis and staging [40]. In a clinical analysis, this study also confirmed that both LINC00265 and LINC00342 were upregulated in osteosarcoma, and the high expression of LINC00265 was closely related to the poor prognosis of osteosarcoma patients. To further analyse the genes associated with osteosarcoma metastasis and vasculogenic mimicry, we also analysed GSE12865 data, which included two groups: osteoblasts and osteosarcoma cells. We compared the genes significantly upregulated in GSE12865 with the genes upregulated in GSE119975, and 70 genes were identified. We believe that these 70 genes are closely related to the growth, metastasis and angiogenesis of osteosarcoma. These 70 genes were analysed using Gene Ontology (GO). The results showed that these genes were primarily enriched in the angiogenesis pathway and the G-protein coupled receptor signalling pathway, both of which belong to the category of biological processes. Five genes were included in the angiogenesis pathway: NRP2, PIK3CG, SAT1, VAV3, and ANGPT2, and PIK3CG was also in the G-protein coupled receptor signalling pathway PIK3CG, SAT1 and VAV3 were chosen for further research. Further clinical analysis studies also demonstrated that PIK3CG, SAT1 and VAV3 were upregulated in osteosarcoma, and their high expression was associated with a poor prognosis. Among these genes, the level of SAT1 and VAV3 was positively correlated with LINC00265. Next, we predicted the miRNAs that might target SAT1 and VAV3 through the website, and the results were overlain with the miRNAs downregulated in GSE12865 and GSE119975. The results showed that there was a common miRNA, miR-382-5p. Further clinical experiments also confirmed that miR-382-5p was underexpressed in osteosarcoma and was significantly associated with a poor prognosis.

It has been found that miR-382-5p is involved in the development and progression of liver cancer and breast cancer [41, 42]. He’s study found that miR-382-5p inhibits cell metastasis and angiogenesis in glioma [43]. In this study, it was confirmed by cell experiments that LINC00265, SAT1 and VAV3 promoted the proliferation, migration, invasion and tube formation of osteosarcoma cells, and LINC00265 promoted SAT1 and VAV3 by targeting miR-382-5p. SAT1 is a polyamine acetyltransferase that is highly expressed in tumours and can serve as a diagnostic marker [44, 45]. In prostate cancer, clinical experiments show that in the progression to advanced metastatic tissues, the level of SAT1 is elevated, suggesting that SAT1 has a role in promoting metastasis [46]. However, the study of Wang shows that upregulation of SAT1 has the effect of inhibiting the progression of liver cancer and colorectal cancer cells [47]. These conflicting results may be due to different causes of the disease, which suggests that SAT1 may have different effects on the cells in different tumours. In osteosarcoma, we found using bioinformatics that SAT1 was related to the poor prognosis of osteosarcoma, and the experiments in vivo and in vitro confirmed that SAT1 had the effects of promoting proliferation and metastasis. VAV3 is an important factor regulating angiogenesis, and VAV3 regulates the Rho/Rac family of GTPases involved in cell growth and movement. Research has shown that the absence of VAV3 inhibits blood vessel growth in tumours and exerts an anti-tumour effect. In recent years, studies have found that VAV3 can be used as a marker for the diagnosis or prognosis of endometrial cancer, colorectal cancer, ovarian cancer and breast cancer [48–51]. One study showed that VAV3 promotes proliferation and epithelial-mesenchymal transition in gastric cancer cells [52]. In addition, Li’s study found that promotion of metastasis by VAV3 can be regulated by miR-499-5p [53]. The promotion of angiogenesis by VAV3 plays an important role in patients with breast cancer metastasis [54]. Combined with this study, we found a ceRNA interaction network, LINC00265-miR-382-5p-SAT1/VAV3, which plays an important role in promoting osteosarcoma metastasis and angiogenesis, and the role of this axis has been verified by animal experiments.

In conclusion, in osteosarcoma, LINC00265 promoted the expression of SAT1 and VAV3 by targeting miR-382-5p and promoted the proliferation, migration, invasion and angiogenesis of osteosarcoma. LINC00265-miR-382-5p-SAT1/VAV3 may be important pathways for the regulation of osteosarcoma metastasis and may affect the prognosis of patients. However, further analysis is needed on the specific mechanism of action and clinical applications.

## MATERIALS AND METHODS

### Bioinformatics analysis

The data related to osteosarcoma and metastasis in the GEO database were selected, and ultimately GSE119975 and GSE12865 were chosen. GSE119975 compared the gene expression levels of osteosarcoma cell lines with and without vasculogenic mimicry. GSE12865 compared limma package; log |FC| > 2 and P <0.01 were used as the threshold. The two analyses were then compared using a Venn diagram to identify the common genes.

The miRNAs related to LINC00265, LINC00342, PIK3CG, SAT1, and VAV3 were predicted using the starBase database, and the predicted results were compared with the miRNAs downregulated in GSE12865.

### Clinical research

A total of 120 osteosarcoma tissues and adjacent tissues were chosen. All samples were diagnosed as osteosarcoma by HE staining. At the time of sample collection, the patient had not received interventions such as chemotherapy and radiotherapy. Quantitative polymerase chain reaction (qPCR) was used to detect LINC00265, LINC00342, PIK3CG, SAT1 and VAV3 expression levels for each case. In addition, the 5-year survival of patients with high or low expression of LINC00265, LINC00342, PIK3CG, SAT1 and VAV3 was compared. Approval was obtained from the ethics committee of the First Hospital of Jilin University.

### Cell culture and transfection

Osteosarcoma cell lines 143B, U2OS, HOS, MG-63, Saos-2 and human osteoblast hFOB 1.19 were purchased from American Type Culture Collection (ATCC, USA) and were grown in RPMI-1640 medium containing 10 % foetal bovine serum (FBS, Thermo Fisher, USA), 50 U/mL penicillin and 50 μg/mL streptomycin (15070063, Thermo Fisher, USA). The database pcDNA3.1 carried human full-length LINC00265, shRNA targeting SAT1/VAV3, and miR-203b-5p mimic/inhibitor, and the corresponding negative control (NC) plasmids were obtained from GenePharma (Shanghai, China). Lipofectamine^TM^ 2000 (Invitrogen, Waltham, USA) was used to transfect 100 pmol shRNA, 50 nM mimic/inhibitor and/or 4 μg plasmid into cells (7 °C, 5 % CO_2_, 48 h). The cells were harvested 48 h after transfection for subsequent experiments.

### qPCR

The total RNA was acquired using TRIzol (Invitrogen, Waltham, USA). For miRNA, complementary DNA was synthesized using a miScript kit (Bio-Rad, California, USA) (7 °C/60 min, 95 °C/5 min, 4°C). A miScript SYBR-Green PCR kit was used for qPCR (95 °C/10 s, 55 °C/30 s, 72 °C/30 s, for 40 cycles) to detect complementary DNA. U6 was used as an endogenous reference for miR-382-5p. For mRNA and lncRNA, reverse transcription (37 °C/15 min, 85°C/5 s) and qPCR (95 °C/5 min, 95 °C/30 s/for 40 cycles, 65°C/45 s) were performed using a PrimeScript-RT kit and a SYBR Premix Ex Taq™ kit (Bio-Rad, California, USA), respectively. The standardized reference was GAPDH. The 2^*−ΔΔCq*^ method was used to analyse the relative expression level of target RNAs [55].

### Western blot

The total protein was extracted using ice-cold RIPA buffer mixed with protease inhibitors (ab65621, Abcam, San Francisco, USA). The protein lysate was separated using SDS-PAGE at 110 V for 100 min and was transferred to PVDF membranes at 90 V for 90 min. The PVDF membranes were blocked in 5 % non-fat milk for 1 h at room temperature, and the antibody (anti-SAT1, ab105220, 20 kD, Abcam, San Francisco, USA; anti-VAV3, ab52938, 98 kD; anti-GAPDH, ab9484, 36 kD) was added at 4°C overnight. The second antibody IgG H&L (HRP) (ab6721, 1:2000) was added to the membrane after washing the membrane with PBST (PBS with 0.2 % Tween 20). A protein blot band was detected using Pierce™ ECL plus a western blotting substrate (Thermo Fisher, Waltham, USA) in ChemiDoc MP (Bio-Rad, California, USA).

### Luciferase assay

The sequences containing the wild-type (WT) or mutated (Mut) region of LINC00265, SAT1 and VAV3 were synthesized by Sangon (Shanghai, China) and inserted into the pGL3 vector (Promega Corporation, Madison, USA). For the luciferase reporter assay, a miR-382-5p mimic or inhibitor and the respective reporter plasmids were transfected into cells using Lipofectamine 2000™ according to the manufacturer’s protocol. After 24 h, the Renilla and firefly luciferase activity was determined using the Dual-Luciferase Reporter Assay System (Promega Corp., Madison, USA) and a luminometer (Infinite 200 PRO NanoQuant, Tecan Group Ltd., Männedorf, Switzerland).

### Cell counting kit 8 (CCK-8) assay

The cells (1 × 10^4^ cells, 100 μL) were seeded in a 96-well plate, and 10 μL per well CCK-8 (Beyotime Institute of Biotechnology, Beijing, China) was then added; the culture was continued for 2 h at 37°C. The absorbance values were measured at 450 nm on a microplate reader (Tecan Infinite M200 Micro Plate Reader; LabX, Switzerland).

### Colony formation assay

A total of 5 × 10^3^ cells were seeded on a 6-well plate with 1 mL medium. After 48 h, cell colonies were fixed with methanol and further stained with 0.5 % crystal violet for 20 min. Colonies were detected under a microscope (Olympus IX71, Tokyo, Japan).

### Wound healing assay

The cells were seeded in a 6-well plate (1 × 10^6^ per well) and cultured with medium until 90 % confluence was achieved in each well. Monolayers of cells were scratched from up to down with the tip of a 200 μL pipette. The monolayers were then washed and further cultured for the next 24 h. Images of monolayers were captured using the inverted microscope. The gaps between the leading edges were measured.

### Transwell assay

A total of 3 × 10^4^ cells were added to the upper chamber of the Transwell apparatus (8-μm, BD Biosciences, CA, USA) with a Matrigel-coated membrane (BD Bioscience, CA, USA) for the invasion assay. The bottom chamber was filled with complete medium supplemented with 10 % FBS. After 48 h, the cells that did not invade through the membrane were swept. The remaining cells were then fixed with 20 % methanol and stained with 0.2 % crystal violet. The cells that invaded into the bottom chamber per field were counted.

### Tube formation assay

An Angiokit™ (TCS cell works, UK) was used to detect tube formation ability in vitro. The experiment was performed in accordance with the manufacturer's instructions. In brief, 1 × 10^4^ cells were seeded on Matrigel and incubated for 6 h. The cells were photographed under a microscope and the cells with a formed tubular structure were counted using Image-Pro Plus 6.0 (Media Cyber Netics, Inc., USA). Five fields of view were counted and averaged.

### Immunohistochemistry (IHC)

The tissue specimens were cut into 4-μm-thick sections. A citrate buffer solution (0.01 mol/L) was used for antigen retrieval and 50 μL of a peroxidase blocking solution was applied to block endogenous peroxidase activity. The stain kit was purchased from Bioss (USA). The primary antibody (anti-SAT1, ab244505; anti-VAV3, ab203315) was added and incubated at 4°C for 12 h. The corresponding secondary antibody was added and incubated at room temperature for 10 min. DAB (100 μL) was added for 5 min, counterstained, and the staining was observed under a microscope (Olympus IX71, Tokyo, Japan).

### Tumour-burden assay

Specific pathogen free (SPF) BALB/c nude mice (4 weeks) were purchased from the animal centre of the Air Force Medical University (Shanghai, China). Cells from lines 143B and U2OS were divided into four groups (n=2): sh-NC+inhibitor-NC, sh-LINC00265+inhibitor-NC, sh-LINC00265+inhibitor and sh-NC+inhibitor. The mice in each group were injected with 1×10^6^ cells. Twenty-eight days after injection, the mice were sacrificed and the tumours were removed to weigh and photograph. The animal experiment protocol was approved by the Animal Experimentation Ethics Committee of The First Hospital of Jilin University.

### Statistical analysis

All analyses were conducted using Prism GraphPad 7.0 software. All variables were reported as the mean ± standard deviation (SD). Comparisons among multiple groups were performed using a one-way analysis of variance (ANOVA). P < 0.05 was considered statistically significant.
